RETRACTED

# Screening of drug candidates against Endothelin-1 to treat hypertension using computational based approaches: Molecular docking and dynamics simulation

**DOI:** 10.1371/journal.pone.0269739

**Published:** 2022-08-18

**Authors:** Israr Fatima, Hamza Ihsan, Muhammad Shareef Masoud, Saeeda Kalsoom, Sidra Aslam, Abdur Rehman, Usman Ali Ashfaq, Muhammad Qasim

**Affiliations:** 1 Department of Bioinformatics & Biotechnology, Government College University Faisalabad-Pakistan, Faisalabad, Pakistan; 2 University of Sargodha Faculty of Medical and Health Sciences Department of Biotechnology, Virtual University of Pakistan, Lahore, Pakistan; 3 Department of Biotechnology, Virtual university of Pakistan, Lahore, Pakistan; Nigde Omer Halisdemir University, TURKEY

## Abstract

Hypertension (HTN) is a major risk factor for cardiovascular and renal diseases, cerebrovascular accidents (CVA) and a prime underlying cause of worldwide morbidity and mortality. Hypertension is a complex condition and a strong interplay of multiple genetic, epigenetic and environmental factors is involved in its etiology. Previous studies showed an association of overexpression of genes with hypertension. Satisfactory control of Blood Pressure (BP) levels is not achieved in a major portion of hypertensive patients who take antihypertensive drugs. Since existing antihypertensive drugs have many severe or irreversible side effects and give rise to further complications like frequent micturition and headaches, dizziness, dry irritating cough, hypoglycemia, GI hemorrhage, impaired left ventricular function, hyperkalemia, Anemia, angioedema and azotemia. There is a need to identify new antihypertensive agents that can inhibit the expression of these overexpressed genes contributing to hypertension. The study was designed to identify drug-able targets against overexpressed genes involved in hypertension to intervene the disease. The structure of the protein encoded by an overexpressed gene Endothelin-1 was retrieved from Protein Database (PDB). A library of five thousand phytochemicals was docked against Endothelin-1. The top four hits against Endothelin-1 protein were selected based on S score and Root Mean Square Deviation (RMSD). S score is a molecular docking score which is used to determine the preferred orientation, binding mode, site of the ligand and binding affinity. RMSD refines value for drug target identification. Absorption, distribution, metabolism, excretion, and toxicity profiling (ADMET) was done. The study provides novel insights into HTN etiology and improves our understanding of BP pathophysiology. These findings help to understand the impact of gene expression on BP regulation. This study might be helpful to develop an antihypertensive drug with a better therapeutic profile and least side effects.

RETRACTED

## 1. Introduction

Hypertension (HTN) is the leading preventable risk factor for cardiovascular diseases (CVD) and renal failure. It is a main cardiovascular risk factor, contributing considerably to cardiovascular disease morbidity and mortality worldwide [1, 2]. Hypertension is defined as a systolic blood pressure ≥140mmHg and/or a diastolic pressure ≥90mmHg. If the parameters are not in accordance then it is considered as one of the most chronic diseases [3]. Ageing and atherosclerosis of arterial walls are also the main cause of HTN. Arteriosclerosis and Vascular stenosis also contribute in elevated blood pressure (BP) [4]. HTN is a complicated disorder influenced by factors such as age, gender, ethnicity, socioeconomic status, education, smoking, BMI, and access to basic healthcare [5]. Multiple studies have found high blood pressure and poor disease control to variables such as age, obesity, low income, poor eating habits, and the lack of basic medical care [6–8].

Maintaining healthy blood pressure (BP) is important to avoid dangerous and life-threatening consequences [9]. Often, HTN is asymptomatic and people don’t visit any doctor which leads to complications [10]. High blood pressure is often known as a silent killer [11]. Although there are generally no symptoms of HTN. Long-term persistence of high blood pressure can damage many organs and cause significant morbidity [12]. Chronic kidney damage due to HTN is the most common cause of stroke and premature death [12, 13]. Endothelin-1 (ET-1) was first characterized as a potent vasoconstrictor and is overexpressed in the vasculature in different models of hypertension, such as deoxycorticosterone acetate-salt rats, Dahl salt-sensitive rats, and stroke-prone spontaneously hypertensive rats [14]. Endothelin-1 is classified as a paracrine or anticrime hormone because over 80% of its secretion by endothelial cells is directed toward neighbouring vascular smooth muscle cells [15]. ET-1’s vascular effects are regulated by the ETA and ETB receptors [16]. The formation of NO and cyclooxygenase derivatives by ETB receptors on endothelial cells causes vasorelaxation [17]. ETB and ETA receptors found on vascular smooth muscle cells, on the other hand, play a role in ET-1’s vasoconstrictor, proliferative, and hypertrophic effects [18].

Metabolic agents (hypoxia) or hormones such as adrenaline, thrombin, vasopressin, angiotensin II (Ang II), insulin, cytokines, and growth factors such as transforming growth factor-1 (TGF-1) can all increase ET-1 development by endothelial cells. Endothelial cells have recently been shown to up-regulate ET-1 activity in response to leptin [19].

RETRACTED

Phytochemicals are non-nutritive chemicals isolated from plants [20]. They can be carbohydrates, polysaccharides, lignin, flavonoids, alkaloids, saponin, steroids or stilbenoids in nature [21]. They are natural and have protective or disease preventive properties like anti-oxidants, anti-bacterial, enzyme stimulators, etc. Making them highly acceptable in the pharmaceutical and food industries [22, 23]. For centuries plants have been the source of treatment for several diseases and many modern medicines have constituents derived from natural sources [24]. These natural compounds are cost-effective and have minimum side effects. Therefore this mode of drug development will lead to an economic treatment regimen [25]. The comparative approach of phytochemicals serves as the best avenue for hunting new cost-effective plants for hypertension [26]. Various natural compounds have been reported to investigate the therapeutic potential of phytochemicals against hypertension [27, 28]. In the current study, the library of 5000 phytochemicals was screened via docking with Endothlien-1. Top resulted compounds Scutellarin & Gentiopicroside were then analyzed by Molecular Dynamic Simulation to check the conformational stability of those candidates for drug designing.

## 2. Materials and methods

### 2.1. Selection of overexpressed Endothelin-1

A detailed and comprehensive literature survey revealed that overexpression of endothelin-1 gene is significantly associated with Hypertension (HTN). The evidence available in literature provided basis for the selection to endothelin-1 gene for its molecular docking.

### 2.2. Structure retrieval & ligand library preparation

The 3D structure of ET-1 protein was retrieved from the protein data bank having PDB ID: 5x93. Endothelin receptor (ETRs) are G protein coupled receptors (GPCR) activated by the vasoactive peptide, endothelin and widely expressed in the vascular endothelium brain and other circulatory organ. This structure revealed the unique binding mode with selected phytochemicals. 5000 phytochemicals were retrieved from PubChem, NPACT, MPD3, ZINC, CHEBL, and ready to dock library was prepared for molecular docking. Docking against Et-1 was used to search the inhibitors using MOE software packages [29]. Sitaxentan is known as an antihypertensive drug, was used as a reference ligand to compare the docking results of phytochemicals.

### 2.3. Protein receptor refinement

The three-dimensional (3D) structure of ET-1 was taken from Protein Data Bank. Removal of water molecules and ligand-receptor are refined. MOE with the following parameters was used to perform 3D protonation and energy minimization; Force Field: MMFF94X+Solvation, Gradient: 0.05, Chiral Constraint Current Geometry. For the docking study, this minimized structure was used as the receptor. 10 poses were selected for the docking in the parameters for findings of best interaction conformations. Reference Drug used before was also docked against the ET-1 to compare the results.

RETRACTED

### 2.4. Analysis of target active binding sites

The site finder tool in Molecular Operating Environment (MOE) software was utilized to find the active sites in the target protein. An active site was defined from the coordinates of the ligand in the original target protein sites.

### 2.5. Molecular docking

The molecular operating environment used to dock 5000 phytochemicals against ligand binding site already reported target binding residues of ET-1 in the Palm I region were done through the MOE site finder tool. The following selected parameters were set for simulation docking: by ligand selected as MBD file of Phytochemicals placement: triangle matcher; re-scoring: London dG: 10; retain: 10: refinement 1: Force field; re-scoring: refinement 2: London dG and retain: 10. Best interacting ligand molecules with targets were screened based on RMSD and Docking score.

### 2.6. Ligand receptor interaction analysis

To have a clear view of receptor-ligand interaction of the best-docked complexes along with the reference drug, The 2D plots of receptor-ligand interactions were analyzed using MOE’s LigX method. It shows a 2D graph of electrostatic interactions, hydrogen bonding, Van der Waals forces, and hydrophobic interactions that are responsible for the affinity in the actively docked pockets of the drug-like molecule. The 3D images of protein inhibitor complexes were generated through MOE [30].

### 2.7. Drug-like properties

All of the finalized phytochemicals were subjected to a drug scan to determine their drug-like properties. As a guideline, Lipinski’s Rule of Five was used. The phytochemical with the highest docking score was then subjected to further selection based on Lipinski’s rule of five (Ro5), with compounds that violated Ro5 being removed. This was simply done by the Molinspiration server for the calculation of their physicochemical properties [31]. The criteria encompass the following molecular properties (MlogP values of less than 5, fewer than 10 H-bond acceptors, less than 5 H-bond donors and molecular weight of fewer than 500 Daltons).

### 2.8. Molecular dynamics simulation

MD simulation is a successful in-*silico* method for studying the dynamic behaviour and stability of protein-ligand complexes under various conditions [32]. Molecular dynamics (MD) simulation of the best ligand poses was performed using the Desmond v3.6 Program to verify the docking performance, as mentioned earlier [33]. In a nutshell, the TIP3P solvent model was used in conjunction with an orthorhombic designed boundary box. By introducing Na + salt, the OPLS-2005 force field was used to counter the process. A hybrid algorithm of gradient descent and LBFGS algorithms was used to decrease the protein-ligand system. After docking, the MD simulation was run at 100 ns on Desmond for early confirmation of the protein-ligand complexes.

RETRACTED

## 3. Results

The database of phytochemicals was docked against ETR protein of hypertension and docked complex were graded based on the straight filter that accounts for four elements including maximum occupancy of binding pocket with east Gibbs free energy, maximum hydrogen bonding interactions and strength of other non-covalent interactions. 100 poses were chosen out of 5000 docked molecules based on the docking score top four ranked docking poses were selected which fulfill the criteria of drug-likeness as shown in **Fig 1**. Reference Drug was **Sitaxentan** used for the comparison of the results in the current study as shown in **Fig 1**.

**Fig 1:** 2D structures of top four selected phytochemicals along with the reference drug.

The results of the top four phytochemicals of ETR protein were selected based on molecular docking score and rmsd-refine values as shown in the **Table 1**.

**Table 1:** The top bioactive phytochemicals interactions along with the docking analysis results.

IDs	Phytochemical Name	Docking score	RMSD value	Interacting Residues
185617	Scutellarin	-18.30	1.41	Asn 158, **Lys 161, Lys 97**
88708	Gentiopicroside	-16.18	1.40	**Lys161, Lys97**
13804	Citicoline	-15.36	1.78	**Lys161, Lys97**
2360	Oxalyldiaminopropionic acid	-10.31	4.05	**Lys161, Lys97**
Reference Drug				
216235	Sitaxentan	-7.40	2.7	**Lys 161, Lys 97**

These selected phytochemicals exhibited their minimum binding energy in the range of -18.30 kcal/mol to -10.31 kcal/mol which was compared to reference drug **sitaxentan** (-7.4 kcal/mol). The minimum binding energy and scoring function of each docked ligand shown in LigX interaction diagram of Scutellarin pocket complex showed strong binding with Asn 158, Lys 161, Lys 97 hydrogen bonds exhibiting a score of -18.30 (kcal/mol) as shown in **Fig 2(A).** The compound Gentiopicroside was revealed to form hydrogen bonds with side chains of residues including Lys 161 and Lys [34] 97 with a binding score of -16.18 (kcal/mol) **Fig 2(B).**

**Fig 2:** Docked scutellarin & Gentiopicroside/Endothlien-1 with ET-1; side chains atoms of Asn 158, Lys 161, Lys 97 making hydrogen bonds. Docked poses of compound highlighting the most active residues of protein’s binding pocket as shown above.

RETRACTED

The compound citicoline was revealed to form hydrogen bonds with side chains of residues including Lys 161, Lys 97, with a binding score of -15.36 kcal/mol, **Fig 3(C).** LigX interaction of Oxalyldiaminopropionic acid showed hydrogen bonding with Lys 161, Lys 97 with a binding score of -10.31(kcal/mol) as shown in **Fig 3(D).**

**Fig 3:** Docked Citicoline & Oxalyldiaminopropionic acid with ET-1; side chains atoms of Lys161, Lys97 making hydrogen bonds. Docked pose of compounds highlighting the most active residues of protein’s binding pocket is shown above.

Our current study results indicated that the inhibiting activity of our compounds was better than the standard drug while targeting the same pocket as shown in **Fig 4**.

**Fig 4:** Reference drug docking complex along interacting residues.

### 3.1. ADMET/Drug scan results

The drug-likeness of the proposed overexpressed proteins of inhibitors was forecast by using the Molinspiration server, based on Lipinski Rules of five. The selected candidate displayed zero and one violations to Lipinski’s rule of five and showed in **Table 2** adequate drug-like properties, i.e.MW.

**Table 2:** Drug candidates exhibiting Lipinski rule of five.

Compounds	Molecular weight (g/mol)	Number of HBA (nON)	Number of HBD (nOHNH)	MLogP
**185617**	459.34	12	4	-2.65
**88708**	354.31	9	2	-3.68
**13804**	487.32	15	4	-6.10
**2360**	174.11	6	2	-5.03
**Reference Drug**				
**216235**	454.91	8	1	3.56

All the selected complexes were subjected for evaluation of pharmacokinetic attributes via the ADMETsar server to confirm the potential of drug likeliness as shown in **Table 3.**

**Table 3:** Drug Candidates exhibiting druglike properties along with the reference drug.

**Compounds**	**185617**	**9848024**	**13804**	**2366**	**Reference Drug**	**216235**
**Blood-Brain Barrier**	Yes	Yes	No	Yes		yes
**Gastro Intestinal Absorption**	low	low	low	low		high
**P-Glycoprotein-substrate**	Substrate	Substrate	Substrate	Non-Substrate		Substrate
**CYP450-1A2-Inhibitor**	No	No	No	No		No
**CYP450-2C9-Inhibitor**	Yes	No	No	No		Yes
**CYP450-2D6-Inhibitor**	No	No	No	No		No
**CYP450-2C19-Inhibitor**	No	No	No	No		No
**CYP450-3A4 Inhibitor**	No	No	No	No		Yes
**Subcellular localization**	Mito-chondria	Mito-chondria	Plasama Membrane	Lysosome		Lysosome

### 3.2. Molecular dynamics simulation

The lead compounds were further investigated by Molecular dynamics using the Desmond System to study the time-dependent divergence of docked protein-ligand complexes up to 100ns after going through docking research, drug-likeness, and ADMET prediction. Basic parameters such as root mean square deviation (RMSD) and protein-ligand interaction were used to estimate the degree of structural changes in complexes and dynamic conduct. Root mean square fluctuation (RMSF), Radius of gyration (Rg) and solvent accessible surface area (SASA) were also calculated. Scutellarin and Gentiopicroside, two phytochemicals derived from top docking findings, formed the much more stable complexes with Endothlien-1 protein. Top two compounds having high Docking score and lower Rmsd value were selected for MD simulation. MD simulation results revealed that the molecule’s energy remains constant throughout the simulation, indicating that the molecule has the stable structure required for simulation.

RETRACTED

#### 3.2.1. Root Mean Square Deviation (RMSD)

The structure vigorous properties of protein/ligand complexes were tested as the backbone RMSDs during the 100 ns MD simulation to track structural and conformational changes. For all frames in the simulation trajectory, the RMSD was determined as the mean distance of the complexes between atoms present in the spine. The RMSD backbone graph of both complexes Scutellarin/Endothlien-1 and Gentiopicroside/Endothlien-1 were shown in **Fig 5**. During the first 30 ns, the RMSD plot of the complex Scutellarin/Endothlien-1 showed good stability after that from 30 to 50 ns it showed a minor variance of 0.5 Å from 50 to 70 ns it showed the variance of 0.3 to 0.4 Å After that the compound showed stability until 95ns as shown in **Fig 5(A)**. The RMSD value of the Gentiopicroside/Endothlien-1 complex, on the other hand, was found to be more stable along the trajectory. Although in Gentiopicroside/Endothlien-1 complex, from 05 to 20 ns and 30 to 40 ns, a minor variation of 0.5 Å was observed. After that complex showed stability up to 85ns from 85 to 90 ns Gentiopicroside/Endothlien-1 complex showed a deviation of 0.3 Å and after that showed stability upto100 ns as Shown in **Fig 5(B)**. For both complexes, the RMSD values steadily increased and remained converged during the simulation period.

**Fig 5:** Detail representation of root mean square deviation plots of protein ligand complex.

#### 3.2.2. Root Mean Square Fluctuation (RMSF)

RMSF metrics were used to examine the flexibility of residues on ligand binding. Common protein flexibility was calculated using RMSF and demonstrates an unpaid parameter to investigate residual protein flexibility throughout the simulation period. Docked complexes RMSF plots are demonstrated in **Fig 6(A)** and **6(B)**. Scutellarin/Endothlien-1 and Gentiopicroside/Endothlien-1 complexes RMSF values were found between a range of 1.2 ± 3Å & 1.2 ± 3.2 Å. Both complexes’ RMSF plots revealed minor differences.

RETRACTED

**Fig 6:** Root mean square fluctuation of docked complexes plots over 100ns.

#### 3.2.3. Radius of gyration (Rg) & Solvent Accessible Surface Area (SASA)

The radius of gyration (Rg) is a mechanism for determining the form and stability of biological molecules during MD time by measuring macromolecule structures. Rg values of both complexes Scutellarin/Endothlien-1 and Gentiopicroside/Endothlien-1 determined during the MD trajectory pose as shown in **Fig 7(E)** and **7(F)**. The Rg values of the complexes Scutellarin/Endothlien-1 and Gentiopicroside/Endothlien-1 obtained by simulation over the time of 100ns were O.46 ± 0.51 and 0.1± 0.96 respectively. Until last the average Rg values of both complexes remained relatively stable. The SASA was used to calculate the water-accessible area of macromolecules. Evaluating the SASA value is an important way to estimate conformational changes caused by complex interactions. For a 100 ns simulation, the approximate average SASA values of the complexes Scutellarin/Endothlien-1 and Gentiopicroside/Endothlien-1 were 0.6 ± 1.5 nm2 & 0.2 ± 0.8 nm2 as shown in **Fig 7(G)** and **7(H)**.

**Fig 7:** The SASA plots of docked complexes over 100 ns MD simulation and the time frame evolution of 100ns against the radius of gyration (Rg) (E & F) (G & H).

#### 3.2.4. Protein-ligand interaction

The ability to predict the binding pocket of docked compounds to the target protein’s binding site requires atomic-level information. The different intermolecular interactions such as hydrogen bonds, water bridges, hydrophobic and ionic interactions were examined over 100 ns of the MD simulation analysis for important mode evaluation. The results indicate that CYS 90, GLN 91, PRO 93, LYS 97ASN 104, SER 108, HIS 150, ACA 154, ASN 158, LYS 161, GLN 181, CYS 255, LEU 257, ASP 274, TYR 281, HIS 340, ARG 343, LYS 346, ASP 368, TYR 369, SER 376 all those amino acids showed strong water bridges. While some amino acid residues like LYS 97, LYS 161, LYS 182, LYS 273, ARG 343 showed compatible ionic bondings with Scutellarin. Some of the hydrophobic interactions with Scutellarin include LYS 182, LYS 273, TRP 336, LEU 339, ARG 343, ILE 372. Scutellarin formed strong hydrogen bonds with the LYS 97, ASN 104, ASN 158, LYS 161, GLN 181, CYS 255, LYS 273 amino acid residues, according to the findings as shown in **Fig 8(I)**. Gentiopicroside formed strong hydrogen bonding with LYS 161, CYS 255, ASP 368 and TYR 369 amino acid residues. Hydrophobic and water bridges includes PRO 88, PRO 89, CYS 90, PRO 93, ILE 94, LYS 161, GLU 165, ASP 166, TRP 167, CYS 174, MET 245, ARG 253, ILE 254, CYS 255, LEU 256, LEU 257, ARG 343, LYS 346, TYR 350, ARG 357, LEU 361, LEU 365, ASP 368, TYR 369 amino acids which showed bonding with the Gentiopicroside as shown in the **Fig 8(J)**.

RETRACTED

**Fig 8:** During 100-ns MD simulation, Endothlien-1 interacts with the compounds as a protein-ligand complex.

## 4. Discussion

In silico research, drug design has been revolutionized by effectively reducing the hustle and overall expense needed by the traditional drug design method. The resources at Level I of drug development have been successfully cut short. New potential drugs and their goals are being discovered and reported in large numbers with the advent of powerful bioinformatics databases, instruments and applications. Due to advances in chemoinformatics, compound libraries are available *In silico* although modern computer techniques are used to screen the properties and drug-like features of those compounds [34].

The current study looked at how phytochemicals from plants interact with the ETR protein. 5000 phytochemicals were tested for their ability to inhibit the overexpressed hypertension ETR protein. Phytochemicals were obtained from a variety of databases. The catalytic triad of overexpressed hypertension ETR protein was docked with phytochemicals to discover their attraction as inhibitors in this research. Only the top conformations from 5000 molecules were chosen after docking based on a minimum S score. Our findings showed that phytochemicals can interact with the active site residues of catalytic triads in a the significant way was cross-checked with standard drug indicate that our reported compounds showed better inhibiting activity as compared to the standard drug.

Our study revealed that four phytochemicals Scutellarin, Gentiopicroside, Citicoline and Oxalyldiaminopropionic acid phytochemicals can interact with the active site residues of catalytic triads in a significant way. The molecular properties and drug-likeness of these four possible compounds were evaluated using ’Lipinski’s Rule of Five. The rule specifies that the compound must have no more than 5 hydrogen bond donors, no more than 10 hydrogen bond acceptors, a molecular mass of fewer than 500 Daltons, and a log coefficient of octanol-water partition P of less than 5.

All executed compounds followed the rule of Lipinski and displayed no desecration. The ADMET profiling of those phytochemicals like Absorption, Delivery, Metabolism, Excretion and Toxicity expected as a drug is further studied. ADMET profiling assessment of top-ranked compounds is the most important for drug development [35]. The numbers of compounds that do not progress through the phase of drug production are due to poor pharmacokinetic properties and toxicity [36]. Early drug discovery is enabled by the development of high-performance and rapid ADMET profiling assays to detect active lead compounds [37]. ADMET profiling of specific lead compounds indicates that all compounds as remedial agents have no side effects on absorption compounds [38]. For several types of models such as P-glycoprotein substrate, BBB penetration, human intestinal absorption, renal organic cation transporter and CaCO2 permeability, ADMET-associated properties of the potential compounds showed positive results which completely support the potential of compounds to act as active compounds. It is found in our studies that all selected flavonoids are non-toxic.

RETRACTED

In this research, we looked for new multi-target drug-like compounds that were derived from plants and had the desired ADME characteristics. To achieve this aim, an in silico structure-based drug design approach was developed to find inhibitors which lead toward four potent common phytochemicals including Scutellarin, Gentiopicroside, Citicoline and Oxalyldiaminopropionic acid. MD Simulation was performed to further evaluate the Scutellarin, Gentiopicroside compounds over a time period of 100 ns. Under the influence of different molecules with binding free energy, the relative importance of amino acids responsible for binding was strengthened. The technique for developing safe and more actual inhibitors for the treatment of HTN was provided by the in-depth description of interrelating remains combined with the vibrant conformations accepted over 100 ns MD simulations of recognized compounds. Based on the binding affinity and score of these phytochemicals were evaluated. The docking analysis identified the most significant residues in terms of binding affinity, namely Lys167 > and Lys61>. The protein-ligand complexes were subjected to MD simulation to further validate the efficacy of the top hit docked compounds. MD simulation is a popular method used in molecular modelling to evaluate the structural modification of the complexes under dynamic conditions. As a result, the stability of docked protein-ligand complexes was assessed using specific parameters such as RMSD, RMSF, Rg, SASA, and protein-ligand interaction in a 100 ns MD simulation using Desmond Package. During the simulation time the compounds Scutellarin and Gentiopicroside, respectively developed good stability in the active site pocket of Endothelin-1, confirming their inhibitory effect. To analyze the structural changes of the protein-ligand complexes, the RMSD values were measured, and both ligand compounds showed minor variations. The versatility of protein chain residues on the ligand-binding site was examined using RMSF plots, and both docked complexes showed small fluctuations during MD trajectories [39]. In addition, the protein-ligand complexes had lower RMSF values, suggesting that they have a secondary structure, such as a helix, which indicates that bound structures are stable. The Rg, which indicates whether the protein-ligand complex will stay unfolded or folded during the simulation phase, revealed that both docked complexes were stably folded during the MD simulation research [40]. The average SASA values projected that the docked complexes would be less exposed to the water solvent during the 100 ns dynamic interactions, implying that they would be more stable. Furthermore, during the 100 ns MD simulation, the protein-ligand interaction analysis showed that numerous intermolecular interactions were involved between Endothelin-1and the two compounds, indicating that the docked complexes were stable [41]. Taking all into account, **Scutellarin** appears to be the best Endothelin-1inhibitor candidate, with a high binding score, conformational stability, and ADMET properties while avoiding the RO5 restriction. The drug candidates were better than standard drug because these candidates were expected to bind selectively to the receptor site on the target to elicit the desired functional response of the target molecule, they were also suitable for clinical testing.

RETRACTED

## 5. Conclusion

*In-silico* molecular docking, research revealed that Scutellarin, Gentiopicroside, Citicoline and Oxalyldiaminopropionic acid phytochemicals extracte had a significant inhibitory effect against the Endothlien-1 protein. At 100 ns dynamic interactions, MD simulation verified the stability of the complexes Scutellarin / Endothlien-1 and Gentiopicroside / Endothlien-1. Moreover, the ADMET and drug-likeness properties of these plant-based natural compounds were favourable. The data generated during the study revealed these active constituents as potential drug targets for the inhibition of upregulated Endothlien-1.”
